# HybridCTrm: Bridging CNN and Transformer for Multimodal Brain Image Segmentation

**DOI:** 10.1155/2021/7467261

**Published:** 2021-10-01

**Authors:** Qixuan Sun, Nianhua Fang, Zhuo Liu, Liang Zhao, Youpeng Wen, Hongxiang Lin

**Affiliations:** ^1^Key Laboratory for Ubiquitous Network and Service Software of Liaoning Province, Dalian, China; ^2^School of Software Technology, Dalian University of Technology, Dalian, China; ^3^The First Affiliated Hospital of Dalian Medical University, Dalian, China

## Abstract

Multimodal medical image segmentation is always a critical problem in medical image segmentation. Traditional deep learning methods utilize fully CNNs for encoding given images, thus leading to deficiency of long-range dependencies and bad generalization performance. Recently, a sequence of Transformer-based methodologies emerges in the field of image processing, which brings great generalization and performance in various tasks. On the other hand, traditional CNNs have their own advantages, such as rapid convergence and local representations. Therefore, we analyze a hybrid multimodal segmentation method based on Transformers and CNNs and propose a novel architecture, HybridCTrm network. We conduct experiments using HybridCTrm on two benchmark datasets and compare with HyperDenseNet, a network based on fully CNNs. Results show that our HybridCTrm outperforms HyperDenseNet on most of the evaluation metrics. Furthermore, we analyze the influence of the depth of Transformer on the performance. Besides, we visualize the results and carefully explore how our hybrid methods improve on segmentations.

## 1. Introduction

Medical image segmentation is an essential area in medical image analysis and is necessary for diagnosis and treatment, which aims to label each pixel in images. Motivated by the recent success of deep learning, researchers in this field have also attempted to apply deep learning-based approaches to medical image segmentation, including U-Nets [1–6] and fully CNNs [7–13]. These methods have achieved superior performance compared to traditional methods in the medical image segmentation task. In order to obtain more accurate segmentation for advanced diagnosis, using multimodal medical images has a growing popularity. Compared with single images, multimodal images help to extract features from different views and bring additional information, contributing to diverse data representation and discriminative power of the network. Previous works usually follow a fully CNN architecture, which suffers from instinctive defects of CNNs. These disadvantages include a deficiency in extracting nonlocal features and bad generalization. With the development of Transformers in language processing, these Transformer-based methods also attract much attention in image processing [14–18], containing classification, detection, and segmentation. These successful applications show the great ability of nonlocal feature extraction for the Transformer-based architecture in images. However, it cannot be directly utilized on multimodal medical image segmentation yet. These works have pretrained with various kinds of images and generated prior knowledge and representations. Pretraining is a self-supervised and auxiliary step and is crucial for the Transformer-based methods since these approaches cannot easily extract enough meaningful representation through the simple task and therefore need transcendental representations from pretraining. Nevertheless, the multimodal medical segmentation task lacks images and therefore cannot follows the pretraining strategy.

In order to tackle these problems, we design a hybrid architecture named HybridCTrm for combining advantages from CNNs and Transformers. Specifically, these networks encode images from CNN and Transformer, two parallel and independent paths, and then integrate representations for decoding and segmentation. In this way, CNNs generate local representations and control gradient descent for rapid convergence, while Transformers extract nonlocal features and avoid overfitting and local optimum in the postperiod of the training. Aiming at fully testing our method, we present two fusion strategies, namely, single-path strategy and multipath strategy, and apply our method on these two different strategies. Experiments and results show that our method can effectively overcome the disadvantages of both CNNs and Transformers, and we show a great improvement in the performance of multimodal medical image segmentation task. Besides, we visualize the results and carefully explore how our hybrid methods improve on segmentations.

## 2. Related Works

### 2.1. Multimodal Medical Image Segmentation Based on CNNs

Multimodal medical image segmentation derives from the medical image segmentation task, both aiming to achieve pixel-level classification for an input image. Traditional medical image segmentation methods generally follow an encoder-decoder architecture, such as U-Net [5] and fully CNN [12]. In these structures, an encoder is usually used to extract features while a decoder is to restore extracted features and output the final segmentation predictions. The U-Net [5] has been widely used for medical image segmentation, consisting of convolution, pooling, and skip-connection. Çiçek et al. [2] extended U-Net architecture to the application of 3D images and proposed 3D U-Net. Milletari et al. [4] proposed V-Net, with residual connections for a deeper network. Similarly, Yu et al. [1] proposed VoxResNet, Lee et al. [3] presented 3DRUNet, and Xiao et al. [6] proposed Res-UNet. In the multimodal medical image segmentation field, researchers generally apply a fully CNN architecture. To effectively employ information from different modalities, Nie et al. [11] proposed a new fully CNN architecture for the multimodal infant brain tissue segmentation. Kamnitsas et al. [10] trained three fully CNNs separately and then averaged the confidence of each network. Chen et al. [7] proposed a dual-pathway fully CNN multimodal brain tumor segmentation network. Wang et al. [13] proposed a cascaded anisotropic convolution network. Dolz et al. [19] proposed a 3D fully CNN based on DenseNets [8].

### 2.2. Image Processing Based on Transformers

Transformers were first applied to natural language processing tasks. Vaswani et al. [20] proposed an attention-pure architecture named Transformer for machine translation and sentence parsing. Devlin et al. [21] proposed BERT, a bidirectional Transformer for two-step training with pretraining and fine-tuning. Brown et al. [22] trained a larger Transformer. Recently, a sequence of Transformer-based methods emerged in the image processing field [14–18]. Among them, Vision Transformer [16] and Detection Transformer [14] are of the most importance. Detection Transformer formulated the detection task as a sequential prediction. Vision Transformer (ViT) cropped an image into a sequence of small patches, which aims to fit the structure of the original Transformer. ViT proved its power on long-range dependencies and showed great performance and therefore was treated as a strong backbone.

## 3. Methodology

### 3.1. Overview Architecture

In multimodal medical image segmentation, the goal is to assign labels for each pixel of the given input images from different modalities. We propose two hybrid architectures for multimodal medical image segmentation as shown in Figure 1. Specifically, we present two models based on two different strategies: single-path strategy and multipath strategy.  Figure 1(a) describes how a single-path strategy works. We take MRI-T1 and MRI-T2 as input modalities. These two modalities *x*^1^, *x*^2^ are combined as a multichannel image *x*^1,2^ and then the image is encoded using convolutions with *m* layers and Transformers with *n* layers. The representations are generated from these two encoders separately and independently and integrated for subsequent decoding. Multipath strategy is quite similar to the single-path one, with the way of input different and Figure 1(b) telling the difference. MRI-T1 (*x*^1^) and MRI-T2 (*x*^2^) are encoded with independent encoders and representations are collected afterward. A multipath network can effectively combine and fully use the information and features from different modalities, while the single-path one focuses more on how different modalities interact with each other. The most key part of our work is that we use Transformers and convolutions as two separate encoders and we will carefully describe the encoders in the rest of the section.

### 3.2. Convolution Encoder

To avoid gradient vanishing and explosion, DenseNets [8] apply skip-connections for directly adding each layer to the follow-up layers. Inspired by the mentioned points, we keep this idea on our convolution encoder.

As shown in Figure 2, a single convolution layer is composed of four parts, batch normalization, PReLU, a 3 *∗* 3 *∗* 3 convolution kernel, and a skip-connection. It is calculated as follows:

(1) $$\begin{array}{c} x_{l}=\left[{\text{Conv}}_{3*3*3}\left(\text{PReLU}\left(\text{BN}\left(x_{l-1}\right)\right)\right.,\;x_{l-1}\right], \end{array}$$

where *x*_*l*_ is the output of the *l*-th layer of convolution and *x*_*l*−1_ is the input of this layer. Particularly, when *l* represents the first layer *l*=1, then *x*_0_ is the input of the images. For multipath strategy, it represents one modality *x*^*i*^ where *i* is not greater than the modality number *n*. Similarly, *x*_0_ represents a combination of input modalities *x*^1,2,…,*n*^ when it comes to the single-path model.

### 3.3. Transformer Encoder

To avoid overfitting and deficiency of nonlocal dependencies generated from fully CNNs, we apply Transformers to encode multimodal images and advance the generalization of the model. Transformers [20] were firstly applied to natural language processing and recently a novel Transformer architecture named Vision Transformer (ViT) [16] was proposed. ViT performed quite well on the image classification task and was quickly accepted as common backbones for image processing.

Inspired by ViT, we modify and apply Transformers for multimodal medical image segmentation as shown in Figure 3. Firstly, we reconstruct a 3D image ${\hat{x}}_{0}\in {\mathbb{R}}^{H\times W\times D\times C}$ into a series of flattened 3D cubes *x*_*p*_ ∈ *ℝ*^*N*×(*P*^2^ · *C*)^, where *N* is the length of the sequence:

(2) $$\begin{array}{c} N=\frac{HW\;D}{P^{2}}, \end{array}$$

where *H*, *W*, *D*, *C* are the height, width, depth, and channel of the origin 3D image ${\hat{x}}_{0}$. For the multipath model, *C*=1 since each input image represents a single modality. For the single-path model, *C* is the modality number *n*. *P* is the size of the cube.

We obtained a patch sequence *x*_*p*_ from the above equations. Transformers apply a constant size *D* for the dimension of each hidden layer. Therefore, we linearly project *x*_*p*_ to *D* dimension and add a position embedding for patch embedding:

(3) $$\begin{array}{c} x_{0}=Wx_{p}+x_{\text{pos}}, \end{array}$$

where *W* is a learnable projection parameter and *x*_pos_ is a learnable position vector. Position embedding *x*_pos_ has the same dimension as *x*_*p*_. It is of great importance in image processing since Transformers do not generate position information and need supplementary inputs. The output, patch embedding *x*_0_, is treated as the input of the first layer of Transformer.

Afterward, *x*_0_ is put into a multilayered Transformer:

(4) $$\begin{array}{c} x_{\text{tmp}}=\text{MHSA}\left(\text{LN}\left(x_{l-1}\right)\right)+x_{l-1},\\ x_{l}==\text{FFN}\left(\text{LN}\left(x_{\text{tmp}}\right)\right)+x_{\text{tmp}}, \end{array}$$

where *x*_*l*_ and *x*_*l*−1_ are the output and input of the *l*-th layer of Transformer encoder. LN (Layer Normalization) is a common design in Transformers and FFN (Feedforward Network) consists of two linear projections and a nonlinear activation function PReLU. MHSA (Multihead Self-Attention) is the crucial part of Transformers and is carefully described in the following.

Different from common Transformers in the image processing field like ViT [16], we modify the position of LN. Xiong et al. [23] proved that the training is more stable when normalization blocks appeared in residual blocks. In our work, multimodal medical image segmentation cannot utilize a pretraining procedure like ViT and thus resulting in much fluctuation when training. Therefore, we apply this modified Transformer architecture to our networks.

MHSA (Multihead Self-Attention) is the core of Transformers and it can be treated as a stack of several simple attention networks. A simple attention mechanism can be calculated as follows:

(5) $$\begin{array}{c} \text{Att}\left(Q,K,V\right)=\text{softmax}\left(\frac{QK^{T}}{\sqrt{d_{k}}}\right)V, \end{array}$$

where the input is copied multiple times and then separated as independent *Q* (queries), *K* (keys), and *V* (values) with their dimension *d*_*q*_, *d*_*k*_, and *d*_*v*_, respectively.

Multiple stacking with simple attention can focus on different representations from different subspaces. Therefore, MHSA projects *Q*, *K*, *V* into different subspaces and conducts attention independently with outputs stacked:

(6) $$\begin{array}{c} \text{MHSA}\left(Q,K,V\right)=\text{Concat}\left({\text{head}}_{1},\ldots ,{\text{head}}_{h}\right)W^{O},\\ \text{where}\;{\text{head}}_{i}=\text{Att}\left(QW_{i}^{Q},KW_{i}^{K},VW_{i}^{V}\right), \end{array}$$

where the projections are parameter matrices *W*_*i*_^*Q*^ ∈ *ℝ*^*d*_model _×*d*_*k*_^, *W*_*i*_^*K*^ ∈ *ℝ*^*d*_model _×*d*_*k*_^, *W*_*i*_^*V*^ ∈ *ℝ*^*d*_model_×*d*_*v*_^, and *W*^*O*^ ∈ *ℝ*^*hd*_*v*_×*d*_model _^. *d*_model_ is the dimension of each hidden layer of Transformers.

### 3.4. Decoder

We use the *l*-th layer output of Transformer encoder *x*_*l*_^trm^ and *k*-th layer output of CNN encoder *x*_*k*_^cnn^ to represent the extracted features from Transformer and CNN. Then, we integrate the features into one matrix *x*^*f*^:

(7) $$\begin{array}{c} x^{f}=x_{l}^{\text{trm}}⊕x_{k}^{\text{cnn}}, \end{array}$$

where ⊕ represents concat operation. Then, feature *x*^*f*^ is sent to a decoder consisting of *l* layers with batch normalization, PReLU, and 1 *∗* 1 *∗* 1 convolution kernel, which is calculated as follows:

(8) xlf=Conv1∗1∗1PReLUBNxl−1f,

and the output of the last layer *x*_*l*_^*f*^ is sent to a Softmax function *p*(*x*) for the final segmentation.

### 3.5. Loss Function and Learning Rate Decay

We apply a common cross-entropy function as our cost function. Let *θ* denote the network parameters and *y*_*s*_^*v*^ the label of pixel *v* in the *s*-th image segment. We optimize the following:

(9) $$\begin{array}{c} J\left(\theta \right)=-\frac{1}{S\cdot V}\sum_{s=1}^{S}\sum_{v=1}^{V}\overset{C}{\underset{c=1}{\sum }}\delta \left(y_{s}^{v}=c\right)\cdot \;\log\;p_{c}^{v}\left(x_{s}\right), \end{array}$$

where *p*_*c*_^*v*^(*x*_*s*_) is the softmax output of the network for pixel *v* and class *c*, when the input segment is *x*_*s*_.

We utilize cosine learning rate decay as our decay strategy:

(10) $$\begin{array}{c} \eta_{t}=\eta_{\min}+\frac{1}{2}\left(\eta_{\max}-\eta_{\min}\right)\left(1+\cos\left(\frac{T_{\text{cur}}}{T_{i}}\pi \right)\right), \end{array}$$

where *η*_*t*_, *η*_max_, *η*_min_ represent learning rate, maximum learning rate, and minimum learning rate, respectively. *T*_cur_ is the iteration number after recurrence and *T*_*i*_ is the current iteration number.

## 4. Results and Discussion

We conduct our experiment on two benchmark datasets, MRBrainS [24] and iSEG-2017 [25]. Both are multimodal medical image segmentation datasets and focus on segmenting three types of brain tissue, including white matter (WM), gray matter (GM), and cerebrospinal fluid (CSF). Between them, MRBrainS is a triple-modal segmentation dataset and iSEG-2017 is a double-modal one.

### 4.1. Experiment Settings

While subvolumes of size 27 × 27 × 27 are considered for training, we use 35 × 35 × 35 nonoverlapping subvolumes during inference, as in [19, 26, 27]. We talked about the cropping and flattening of a given image in the previous sections. Among them, *P* is the size of a cube and is crucial for computation costs and performance. When *P*=1, MHSA can calculate with each pixel. However, it will cause high computation costs and go beyond limited GPU resources. With a big *P*, Transformers cannot effectively capture features. Based on these two points, we set *P*=3. For Transformers, we set the head to be 4, hidden dimension to be 128, and depth to be 4 according to the experiment performance. To initialize the weights of the convolution path, we adopt the strategy proposed in [28], which yields fast convergence for very deep architectures. In this strategy, a zero-mean Gaussian distribution of standard deviation $\sqrt{2/n_{l}}$ is used to initialize the weights in layer *l*, where *n*_*l*_ denotes the number of connections to the units in that layer. The initial learning rate (*η*_max_) is set to be 1*e* − 4. For cosine decay, *η*_min_ is 5*e* − 5 and *T*_cur_ is 50. Considering limited GPU resources, we set the batch size to be 32.

We compare our modal with several fully CNN-based architectures, including fCNN [12], CNN_small_ [27], CNN_small_ − MS [27], and HyperDenseNet [19]. fCNN [12] was the first method that applied CNNs to segmentation tasks. Then, Dolz et al. [27] set a smaller kernel for convolutions and presented two kinds of methods including traditional one and multiscaled one. HyperDenseNet [19] was a commonly used fCNN-based method in multimodal image segmentation tasks. These models can be effectively compared with our hybrid model, HybridCTrm. To fairly compare with baselines, we conduct experiments with two strategies, single-path and multipath separately, and set a postfix, like -Multi and -Single, for each method.

We apply Dice Similarity Coefficient (DSC) as evaluation metrics, a common method for segmentation evaluation [19, 26, 27]:

(11) $$\begin{array}{c} \text{DSC}=\frac{2\text{TP}}{\text{FP}+2\text{TP}+\text{FN}}. \end{array}$$

## 5. Results on MRBrainS

We apply leave-one-out-cross-validation for a five-sample dataset, MRBrainS, that is, four samples for training and one for testing. We report DSC on three tissues (CSF, GM, and WM) and their average.

### 5.1. Main Results

Table 1 shows general results of our method and baselines on MRBrainS and the highest score on each column is bold.

A general view shows that our hybrid network achieves the highest score on each metric. To have a clear comparison, we firstly compare two simple-path models. We mostly compare our method with HyperDenseNet, since this model performs the best among CNN-based architectures on each strategy. Compared with HyperDenseNet-Single, HybridCTrm improves by about 3%, 1%, and 26% in WM, GM, and CSF, respectively. At the same time, the average score outperformance is 10%. For multipath models, HybridCTrm-Multi improves by 4% and 18% on CSF and WM tissue compared with HyperDenseNet-Multi. Then, we focus on the performance of the same model on different strategies. For segmenting GM and CSF tissue, multipath strategy is more fitting, while single-path one performs better on WM. This may infer that, for segmenting GM and CSF information from different modalities, it is needed to encode independently first and then integrate with each other, while for WM it is the opposite.

### 5.2. Analysis of Hyperparameters

In order to better analyze the influence of Transformers on performance, we conduct experiments with different depths of Transformers settings.

Figure 4 shows how depth influences performance on single-path and multipath models. For HybridCTrm-Single, the average DSC reaches the peak at the depth of 4. The curve increases firstly and then drops with the increase of depth from 1 to 5. For HybridCTrm-Multi, the peak reaches the depth of 5 and the trendy of the curve is quite similar, from rising to declining. This similar trend is probably because different depths capture different representations and a suitable depth can extract the most effective information for segmentation.

### 5.3. Ablation Study

Our hybrid architecture consists of a CNN encoder and Transformer encoder to capture local and nonlocal features for segmentation. To research how CNN and Transformer branches influence our hybrid model, we conduct an ablation study. As shown in Table 2, we separate the CNN branch and Transformer branch, respectively, based on the single-path model and multipath model. After removing the CNN branch, the mean DSC drops by about 48% and 46% for single and multistrategy, respectively, while it drops by about 16% and 13% with removing the Transformer branch. It shows that compared with the Transformer branch, the CNN branch is more important because nonlocal features extracted by the Transformer encoder play an auxiliary role in the segmentation.

### 5.4. Auxiliary Experiments with Dual Modality

To further analyze the importance of segmentation of different modalities, we choose two modalities and conduct auxiliary experiments with dual modality.

As shown in Table 3, the results of three modalities perform better compared with the two modalities. However, a careful comparison clearly shows that the results based on the T1 and T2-FLAIR modalities have the lowest performance degradation (only 2%–3%), indicating a strong complementarity between these two modalities. The other two modal combinations, T1 and T1-IR, and T1-IR and T2-FLAIR, show significant performance degradation (10%–13%), indicating that the T1-IR modality does not bring more information. A further comparison of the performance of CSF, GM, and WM tissues shows that the performance of the combination of T1 and T2-FLAIR on CSF and WM is comparable to that of the three modalities under the corresponding strategies. And the former is even 0.6% higher than the latter under the multipath strategy, which indicates that the information in these two modalities is sufficient to segment the CSF and WM tissues. This indicates that the information in these two modalities is sufficient to segment CSF and WM tissues. On the contrary, the performance of segmentation on GM tissues is best only when the information in the three modalities is complete, and there is a 5%–6% degradation in the results of the other two modalities.

### 5.5. Results on iSEG-2017

We divide the iSEG-2017 dataset with 10 samples into a training set (train), a development set (dev), and a test set (test) in the ratio of 8 : 1 : 1. The detailed results are presented in Table 4, and the maximum value of each item is bold.

### 5.6. Main Results

First, our HybridCTrm network outperforms in seven out of eight metrics among all these methods. Compared with HyperDenseNet-Single, HybridCTrm-Single outperforms in all metrics. This is because the information in the single-path strategy is integrated at the beginning, and the Transformer structure can fully model this complex information. In the multipath strategy, HybridCTrm-Multi also outperforms HyperDenseNet-Multi in seven metrics, further validating the modeling capability of Transformer. However, the gain is not as great as the single-path model. This is probably because the information content of each individual modality is small, so the Transformer cannot learn enough features like the CNN with strong inductive bias.

### 5.7. Analysis of Generalization and Stability

Having already concluded that hybrid structure-based models work better than pure fCNN models, we are also concerned about the stability and generalization performance of the models.

Figure 5 shows the performance of the two models on the development set and the validation set under the two strategies after every 5 epochs. The left panel shows the performance of the two models under the single-path strategy. The red line represents HybridCTrm and the blue line represents HyperDenseNet, while the solid line represents the performance on the development set and the dashed line represents that on the test set. It can be seen that HybridCTrm is always better than HyperDenseNet in both the early and late stages of model training, and it can be concluded that the hybrid structure can converge more rapidly than the fCNN structure under the single-path strategy. Meanwhile, in the middle and late stages of model training, it can be found that the training based on HyperDenseNet is not stable, and sometimes there is a sudden drop, while HybridCTrm is more stable. For the multipath strategy, HybridCTrm is significantly better than HyperDenseNet in the early and middle training stages, indicating that the former can provide faster convergence under the multipath strategy. The stability of HyperDenseNet is slightly better than that of HybridCTrm in the middle and late stages of training. This may be because the model has learned enough good features in the middle and late stages of training, and further learning is much difficult for Transformers to utilize each modal information separately. Therefore, there may be some bad features in the layers of the Transformer, resulting in a decrease in the stability of the model. For HyperDenseNet, the features of the CNN are more stable and therefore do not produce large fluctuations. On the other hand, the slight instability in the later stages also allows the model to learn more randomly and avoid falling into local minima that lead to poor global generalization performance.

### 5.8. Visualization

To further explore the advantages and disadvantages of different models and preferences for segmentation content, segmentation results from a partial test set are shown for visual analysis.

Figure 6(a) shows a segmented 2D section. In the frame region, the CSF tissue (blue part) shows a striped distribution, while HyperDenseNet performs poorly on CSF under both the single-path strategy and multipath strategy. On the contrary, HybridCTrm performs well in CSF segmentation, especially in the single-path strategy, where the continuous bar distribution of CSF is reflected. For GM tissue (green part), HyperDenseNet misclassifies a large part of the gray matter as WM (yellow part) and generates a lot of “adhesions” in the WM region. The HybridCTrm, on the other hand, has a good performance on the GM and better reflects the contour structure, indicating that the hybrid structure fully exploits the long-distance dependence.

Figure 6(b) shows another segmentation profile, in which we focus on the forebrain part: the boxed area in the figure. We can see that there is a clear section of the GM pathway in the target region, which is missegmented as WM tissue in the HyperDenseNet, but better segmented in the HybridCTrm. Meanwhile, on the rightmost side of the box, there is a small piece of CSF tissue, which is not segmented at all under the HyperDenseNet-Single and is minimally segmented under the HyperDenseNet-Multi. In the HybridCTrm, this part is also well segmented.

## 6. Conclusion

This paper discusses the application of hybrid networks based on CNNs and Transformers in the field of multimodal medical segmentation and proposes a novel multimodal medical segmentation architecture, HybridCTrm. Two multimodal segmentation strategies are proposed, namely, single-path strategy and multipath strategy. In the experiment, the HybridCTrm architecture is tested on two benchmark datasets under single-path and multipath strategies and compared with HyperDenseNet, an architecture based entirely on the fully CNNs. HybridCTrm outperforms HyperDenseNet in most of the metrics.

## Figures and Tables

**Figure 1:** Two hybrid architectures. (a) Hybrid Convolution-Transformer model with a single path. (b) Hybrid Convolution-Transformer model with multipath.

**Figure 2:** Convolution encoder.

**Figure 3:** Transformer encoder.

**Figure 4:** Performances of different depths of Transformers.

**Figure 5:** DSC curve.

**Figure 6:** Visualization.

**Table 1:** Main results on MRBrainS.

	CSF	GM	WM	Mean
fCNN-Single [12]	52.55	73.62	74.82	66.99
fCNN-Multi [12]	67.03	80.59	62.50	70.04
CNN_small_-Single [27]	58.49	74.66	71.31	68.16
CNN_small_-Multi [27]	62.26	81.93	81.67	75.29
CNN_small_-MS-Single [27]	42.88	70.02	80.66	64.52
CNN_small_-MS-Multi [27]	64.08	82.09	59.23	68.46
HyperDenseNet-Single [19]	49.12	84.14	85.85	73.04
HyperDenseNet-Multi [19]	72.90	85.06	70.64	76.20
HybridCTrm-Single	75.09	85.30	88.54	82.98
HybridCTrm-Multi	76.53	85.52	88.37	83.47

**Table 2:** Ablation study.

	CSF	GM	WM	Mean
HybridCTrm-Single	75.09	85.30	88.54	82.98
W/o CNN branch	30.39	44.91	54.64	43.31
W/o Transformer branch	56.18	84.11	68.64	69.64
HybridCTrm-Multi	76.53	85.52	88.37	83.47
W/o CNN branch	32.72	50.36	52.48	45.19
W/o Transformer branch	75.32	81.48	62.03	72.95

**Table 3:** Auxiliary results with dual modality.

	Modality	CSF	GM	WM	Mean
HybridCTrm-Single	T1, T1-IR	53.89	79.75	81.88	71.84
HybridCTrm-Single	T1, T2-FLAIR	75.09	79.88	87.92	80.96
HybridCTrm-Single	T2-FLAIR, T1-IR	56.13	79.78	69.94	68.61
HybridCTrm-Single	3 modalities	75.09	85.30	88.54	82.98
HybridCTrm-Multi	T1, T1-IR	69.88	78.17	71.68	73.25
HybridCTrm-Multi	T1, T2-FLAIR	74.07	78.97	88.89	80.64
HybridCTrm-Multi	T2-FLAIR, T1-IR	68.54	80.20	64.17	70.97
HybridCTrm-Multi	3 modalities	76.53	85.52	88.37	83.47

**Table 4:** Main results on iSeg-2017.

	Dev				Test			
	CSF	GM	WM	Mean	CSF	GM	WM	Mean
fCNN-Single [12]	89.21	86.56	78.31	84.55	85.66	83.13	82.84	83.87
fCNN-Multi [12]	89.98	85.35	78.31	84.55	85.66	83.13	82.84	83.87
CNN_small_-Single [27]	92.42	89.00	81.74	87.72	88.59	85.47	83.47	85.84
CNN_small_-Multi [27]	93.13	89.24	82.73	88.36	88.92	85.85	85.26	86.68
CNN_small_-MS-Single [27]	92.75	89.59	82.98	88.44	88.69	85.95	84.36	86.33
CNN_small_-MS-Multi [27]	92.81	89.77	82.01	88.20	89.35	85.71	83.09	86.05
HyperDenseNet-Single [19]	92.24	88.58	81.18	87.33	88.59	85.40	83.92	85.97
HyperDenseNet-Multi [19]	92.99	89.39	83.24	88.54	88.85	85.87	85.35	86.69
HybridCTrm-Single	93.38	88.66	82.21	88.08	89.24	85.90	85.11	86.75
HybridCTrm-Multi	93.46	90.26	83.71	89.14	89.75	86.40	85.34	87.16

## Data Availability

The data used to support the findings of this study are available from the corresponding author upon request.
